# Patient engagement and patient support programs in allergy immunotherapy: a call to action for improving long-term adherence

**DOI:** 10.1186/s13223-016-0140-2

**Published:** 2016-07-29

**Authors:** Pascal Demoly, Giovanni Passalacqua, Oliver Pfaar, Joaquin Sastre, Ulrich Wahn

**Affiliations:** 1 Department of Pulmonology, Division of Allergy, Hôpital Arnaud de Villeneuve, University Hospital of Montpellier, Montpellier, France; 2 Sorbonne Universités, UPMC Paris 06, UMR-S 1136, IPLESP, Equipe EPAR, Paris, France; 3 Allergy and Respiratory Diseases, IRCCS San Martino-IST, University of Genoa, Genoa, Italy; 4 Center for Rhinology and Allergology, Wiesbaden, Germany; 5 Department of Otorhinolaryngology, Head and Neck Surgery, Universitätsmedizin Mannheim, Medical Faculty Mannheim, Heidelberg University, Mannheim, Germany; 6 Allergy Department, Fundación Jimenez Díaz, Madrid, Spain; 7 CIBERES, Instituto de Salud Carlos III, Universidad Autonoma de Madrid, Madrid, Spain; 8 Department of Pediatric Pulmonology and Immunology, Charité Virchow-Klinikum, Humboldt University, Berlin, Germany

**Keywords:** Adherence, Patient engagement, Patient support program, Allergy immunotherapy

## Abstract

Allergy immunotherapy (AIT) is acknowledged to produce beneficial mid- and long-term clinical and immunologic effects and increased quality of life in patients with allergic respiratory diseases (such as allergic rhinoconjunctivitis and allergic asthma). However, poor adherence to AIT (due to intentional and/or non-intentional factors) is still a barrier to achieving these benefits. There is an urgent need for patient support programs (PSPs) that encompass communication, educational and motivational components. In the field of AIT, a PSP should be capable of (1) improving adherence, (2) boosting patient engagement, (3) explaining how AIT differs from pharmacological allergy treatments; (4) increasing health literacy about chronic, progressive, immunoglobulin-E-mediated immune diseases, (5) helping the patient to understand and manage local or systemic adverse events, and (6) providing and/or predicting local data on aeroallergen levels. We reviewed the literature in this field and have identified a number of practical issues to be addressed when implementing a PSP for AIT: the measurement of adherence, the choice of technologies, reminders, communication channels and content, the use of “push” messaging and social networks, interactivity, and the involvement of caregivers and patient leaders. A key issue is “hi-tech” (i.e. approaches based mainly on information technology) vs. “hi-touch” (based mainly on interaction with humans, i.e. family members, patient mentors and healthcare professionals). We conclude that multistakeholder PSPs (combining patient-, provider and society-based actions) must now be developed and tested with a view to increasing adherence, efficacy and safety in the field of AIT.

## Background

Allergy immunotherapy (AIT, either sublingual or subcutaneous) is acknowledged to have beneficial mid- and long-term clinical and immunologic effects on patients with allergic respiratory diseases (such as allergic rhinoconjunctivitis and allergic asthma). In particular, those effects may persist for several years after discontinuation [1–4]. Indeed, long-term efficacy and sustained (post-treatment) efficacy are important parameters in the regulatory approval of AIT formulations in Europe [5]. Even though AIT has a relatively short (intra-season) onset of action [6] for symptom relief, multi-season or multi-year administration of AIT is required to achieve a long-lasting, disease-modifying effects. Poor adherence to long-term AIT (as with other chronic treatments) is thus a barrier to obtaining allergen tolerance, symptom relief and improved quality of life (QoL).

## Review

### Adherence to long-term treatment: a key reason for trying to boost patient engagement

Although progress in technology and medicine offers great opportunities for healthy living, successful outcomes are increasingly reliant on the patient’s active participation in his/her treatment. However, one of the main problems in modern medicine—especially in the field of chronic disease—is patient adherence, defined by the World Health Organization as *“the extent to which a person’s behavior—taking a medication, following a diet or executing lifestyle changes—corresponds with agreed recommendations from a healthcare provider”* [7]. In a quote attributed to the former US Surgeon General Dr. C. Everett Koop, “*drugs don’t work in patients who don’t take them*”.

Adherence can be broken down into several stages (Fig. 1): (1) initiation (also referred to as acceptance), (2) implementation (also referred to as compliance, i.e. the proportion of the recommended doses of medication actually taken by the patient) and (3) persistence (i.e. not discontinuing the treatment before the end of the recommended period) [7–9]. There are many intentional or non-intentional reasons why a patient may fail to take his/her medication or not follow other healthcare measures prescribed by a physician (Table 1) [10, 11]. However, most (but not all) studies of non-adherence in chronic disease suggest that non-intentional reasons predominate—mainly “I simply forgot” and variants of the latter [12, 13]. In intentional non-adherence, patients often irrationally consider that the risks associated with adherence are greater than the risks associated with non-adherence (Table 1).

**Fig. 1:** A schematic diagram of the components of adherence. Adapted from [6–8]

**Table 1:** Barriers to good adherence and patient engagement [6–14] and the corresponding interventions

Factors in poor adherence and examples	Interventions for patient support programs
*Intentional factors*	
***Fear and experience of side effects*** *The patient has experienced or fears experiencing side effects and thus avoids taking the medication*	Explanation and coaching by healthcare professionals (patient empowerment)
	Collaborative care and raised awareness of AIT
***Lack of perceived efficacy*** *The patient considers that the medication is not “working” and is of no value*	Individual patient coaching
	Explanation and coaching by healthcare professionals (patient empowerment)
	Collaborative care and raised awareness of AIT
***High perceived efficacy*** *The patient considers that the medication has done its job and can thus be discontinued*	Individual patient coaching
	Coaching by healthcare professionals (patient empowerment)
	Collaborative care and raised awareness of AIT
***Financial issues*** *The patient considers that he/she can save money by reducing the number of doses or the duration of treatment*	Point-of-care cost reduction
***Social issues and lack of convenience*** *The patient is embarrassed to take his/her medication when outside the home setting (for AIT normally administered at home) or fails to renew or collect a prescription due to travel/cost issues*	Easy-to-administer formulations
	Patient mentors
	Explanation and coaching by healthcare professionals (patient empowerment)
***Psychological factors*** *The patient does not accept that he/she is really ill (denial of the disease), and so not taking the medication helps him/her to think less about the disease*	Explanation and coaching by healthcare professionals (patient empowerment)
	Collaborative care and raised awareness of AIT
*Non*-*intentional factors*	
***Forgetfulness*** *The patient forgets to take his/her medication. Forgetfulness can be accentuated by a number of lifestyle and health*-*related factors (travel, age, co*-*morbidities, social activities* etc*.)*	Reminders sent by: telephone (automated or human), text messages, e-mail, social networks, electronic pillboxes.
	Patient mentors
	Individual patient counselling
***Poor physician-patient communication and/or poor health literacy*** *The patient does not understand the dosing instructions and/or does not how to resume treatment after interruption*	Clearer product information sheets
	Simplified but safe regimens for resumption after interruption
	Patient mentors
	Explanation and coaching by healthcare professionals (patient empowerment)
	Collaborative care and raised awareness of AIT
***Unscheduled travel or school/work commitments*** *The patient has to travel or change his/her daily routine unexpectedly, which interferes with taking medication*	Easy-to-administer formulations
	Reminders sent by: telephone (automated or human), text messages, e-mail, social networks, electronic pillboxes
***Poor stock management*** *The patient fails to anticipate the need to renew a prescription and therefore runs out of medication*	Reminders sent by: telephone (automated or human), text messages, e-mail, social networks, electronic pillboxes
	Individual patient coaching

### Levels of adherence in patients on AIT

It has been estimated that the compliance rate for drug therapy of chronic disease is barely over 50 % [7]; most of these data have come from studies of patients with diabetes, chronic kidney disease, neurologic disorders, cardiovascular disease or AIDS. In the literature on AIT, the compliance component of adherence ranges from around 25 % to over 90 % [14]. In a recent Italian study of sales data provided by two major manufacturers, more than 50 % of patients discontinued sublingual allergy immunotherapy (SLIT) during the first year, and only 13 % were still on treatment in the second year. This shortfall was independent of the allergen source, administration regimen and, in part, reimbursement status [15]. A German retrospective analysis of renewal rates for grass pollen AIT found that 49 and 64 % of patients did not renew their SLIT or SCIT prescription, respectively, over 2 years [16]. Hence, increasing the adherence rate may be an important way of improving safety, efficacy, quality of life (QoL) and other patient-related outcomes in AIT.

### Key factors in improving adherence rates

A multitude of organizational, educational and technological interventions have been developed or proposed with a view to improving adherence and patient outcomes. In a Cochrane review, Haynes et al. [17] reported that only 26 out of 58 interventions in 49 randomized clinical trials were associated with improved adherence, and that almost all of the interventions with long-term efficacy were complex and multifactorial. Furthermore, it appears to be impossible to predict which interventions will or will not work in a particular setting and over a given timeframe. Behavioral interventions for enhancing medication adherence (when behavioral counselling is directly offered to patients by specifically trained health care professionals) have shown contradictory results [18]. Unfortunately, even the most successful interventions did not produce large improvements in adherence.

Patient education, health literacy, patient-centered care, patient-centered communication, patient activation and patient engagement are related but non-identical approaches that can potentially improve adherence. Firstly, patient education has been variously defined as “*any set of planned educational activities designed to improve patients’ health behaviors and health status*” [19] and “*a process of assisting consumers of health care to learn how to incorporate health*-*related behaviors (i.e., knowledge, skills and/or attitudes) into everyday life with the purpose of achieving the goal of optimal health”* [20]. Secondly, health literacy is defined by the US Institute of Medicine of the National Academies as “*the degree to which individuals have the capacity to obtain, process, and understand basic health information needed to make appropriate health decisions*” [21]. Low health literacy is associated with poor adherence and poor outcomes [22–24]. However, most programs based on health education, information, literacy or numeracy alone have failed to improve adherence, even though they do improve the level of knowledge about disease [16, 25].

Lastly, patient engagement—described as “*the blockbuster drug of the century*” [26]—has been defined as “*actions [that] individuals must make to obtain the greatest benefit from the health care services available to them*” by the Center for Advancing Health [27] and “*the involvement in their own care by individuals (and others they designate to engage on their behalf), with the goal that they make competent, well*-*informed decisions about their health and health care and take action to support those decisions*” by the Agency for Healthcare Research and Quality [28]. Both these definitions emphasize that even a well-informed, health-literate patient must also be personally committed, motivated and pro-active if he/she is to help prevent, manage and treat his/her disease. It has been reported that in patients with chronic metabolic diseases, empowerment-based self-management interventions have stronger, long-lasting effects than conventional self-management or education, although adherence has not always been assessed in these studies [29–31]. Furthermore, the time that healthcare professionals can dedicate to allergic patients (and their parents, when considering pediatric patients) in the office may modulate the above-mentioned educational and psychological factors. For example, Rolinck-Werninghaus et al. [32] reported that an individually tailored nurse consultation for parents of children with atopic dermatitis was associated with significant benefits in terms of reduced disease severity and confidence in dealing with the disease. Group educational programs were particularly effective in parents with poor coping abilities at baseline [33].

### Patient engagement and patient support programs (PSPs) in the field of respiratory allergies and AIT

Patient engagement must be kindled and maintained. PSPs (including communication, educational and motivational components) are intended to boost patient engagement, improve adherence (initiation, compliance and persistence), help patients understand and manage their disease, improve QoL and facilitate patient-physician communication, concordance and trust.

In the field of AIT, a PSP will have additional, specific objectives:

- Explain the benefits of AIT and how it differs from other allergy treatments: the disease-modifying mode of action vs. symptomatic medication, short- and long-term benefits of AIT, modes of administration, the recommended duration of treatment (3–5 years), the onset of action of AIT (as early as the first season, within 1–4 months of initiation [6]), reduction in the need for pharmacotherapy, and possible prevention of the progression of the allergic disease such as secondary/tertiary prevention regarding the development of asthma [4, 34].
- Increase health literacy about allergic disease (from the diagnosis onwards, if possible), with a focus on chronic, progressive, immunoglobulin-E-mediated immune diseases with health, work and QoL consequences.
- Help to understand and manage local or systemic adverse events and those related to the administration route, whether SLIT or subcutaneous allergy immunotherapy (SCIT).
- Improve adherence year after year or season after season, in order to obtain the disease-modifying benefits of AIT.
- Provide data on and/or predict aeroallergen and pollutant levels on a local basis (for a patient’s place of residence or when travelling), with customized alerts for specified allergen sources. This is essential in pollen-induced allergies, due to the well-known variability of pollen seasons as a function of geographic location and climate. Prediction of the start of a pollen season is less useful in patients following a perennial AIT regimen or a pre- and co-seasonal regimen than is initiated before the start of the season. However, confirmation of the end of a pollen season may be more valuable for highlighting the end date for co-seasonal administration.

Allergists are clearly moving towards patient-centered care and PSPs, as illustrated by the new MASK-rhinitis IT tool (developed as part of the European Innovation Partnership on Active and Healthy Ageing) for diagnosing, stratifying and managing patients with AR and assessing treatment efficacy [35]. The MASK-rhinitis smartphone application for the patient combines e-Allergy screening (for early online diagnosis of allergy and asthma), the daily rating of rhinitis symptoms on a visual analogue scale and an assessment of disease control using the control of allergic rhinitis and asthma test. It is interfaced with a clinical decision support system based on the widely used allergic rhinitis in asthma guidelines [36]. With the rapid growth of mobile Internet use, smartphone apps are inevitably going to be key components of PSPs.

The field of asthma (a condition that is generally but not always allergic) may provide valuable insights for PSPs in AIT of allergic respiratory diseases. Over the last few decades, intense effort has been devoted worldwide to delivering and promoting asthma education, self-management and personal action plans. By way of an example, a recent study has shown that self-monitoring, individualized asthma action plans, information about assessments and correct use of an inhaler do increase adherence and provide clinically useful data on disease control [37]. In another study, an intervention based on a “physician on call patient engagement trial” mobile phone application was associated with improvements in activity, productivity, disease control, disease perception and emotion, although adherence was not assessed [38]. However, systematic reviews of this aspect revealed the absence of a clear clinical trial-based evidence in favor of these asthma interventions. In Coffman et al.’s US-based meta-analysis of the effects of pediatric asthma education on hospitalizations, emergency department visits, and urgent physician visits, 37 trials met the meta-analysis’ inclusion criteria [39]. The researchers concluded that although pediatric asthma education reduced the mean number of hospitalizations and emergency department visits and the likelihood of an emergency department visit, there was no significant effect on the likelihood of hospitalization in general or the mean number of urgent physician visits. Similarly, in a meta-analysis of 37 studies, Pinnock et al. [40] concluded that only “whole systems approaches” that explicitly and simultaneously addressed patient-, professional- and organization-related factors were associated with consistent improvements in clinical outcomes in asthma, although adherence per se was rarely studies. This approach typically combined (1) direct patient coaching, free resources, patient mentors and/or group activities, (2) continuing professional education and training for specialists and/or primary care physicians, and (3) local and/or national health promotion and awareness programs [40].

### A call to action for PSPs in the field of AIT

A number of practical questions and choices must be considered when implementing a PSP for AIT. We encourage researchers, physicians, other healthcare professionals, learned societies, medical associations and patient organizations to explore and refine the following points.

- Levels of adherence should be measured as soon as a patient has been prescribed AIT and then on a regular basis thereafter. Both patients and physicians should be able to display data on changes over time in adherence and engagement. Validated tools exist, such as the 4- or 8-item Morisky Medication Adherence Scale [41]. The PSP interface could also be used to assess disease control in allergic rhinitis or asthma [42, 43]. Ideally, a PSP should be able to identify particular barriers to adherence (see Table 1), characterize non-adherence profiles (poor dosage vs. poor persistence, for example) and adapt actions and content accordingly. For example, a patient suffering from forgetfulness could be invited to view a short video giving behavioral tips on improving self-organization. A PSP should also be able to rapidly detect patients with special communication needs.
- *Technological choices* Modern technology enables the interactive, mass dissemination of customized information. However, the application of technology per se is not a panacea for engagement and adherence; “hi-tech” must be balanced against “hi-touch”—the maintenance of a close personal connection. Mistry et al. [44] have stated that there are too few high-quality studies to reliably assess the effectiveness of technology-mediated interventions; of 38 studies reviewed, 24 did not find significant effects on both adherence and clinical outcomes. By way of an example, Alesina et al. [45] recently studied the use of an electronic tablet container (the Memozax) with a programmable daily sound alarm in 261 patients taking a timothy grass pollen sublingual AIT tablet in Italy. The patients were randomized 1:1 to use of the device or not. After 1 year, the compliance rate in the Memozax group was slightly higher (91.7 %) than that in the non-Memozax group (90.3 %) but this difference was not statistically significant. In general, there is a lack of robust, clinical trial data on the efficacy of health information technology tools in the self-management of respiratory disease. Easy access to the Internet and the ease with which apps can be created have disadvantages, too; the same group’s review of 103 apps for asthma in English found that none combined reliable, comprehensive patient information with supportive tools for self-management [46]. In a recent Cochrane Collaboration review, the same group searched for randomized controlled trials on the clinical effectiveness, cost-effectiveness and feasibility of smartphone and tablet apps in the self-management of individuals with asthma. Only two trials (totaling 408 participants) met the inclusion criteria, and neither found a significant effect on adherence [47].
- *Reminders, communication channels and content* A PSP designed to enhance adherence is likely to feature prominent reminders to take medications, refill prescriptions or contact a healthcare professional. These reminders may be based on phone calls, text messages, e-mail messages, pagers, interactive voice response systems, video calls, “smart” electronic medication containers, or combinations thereof. Furthermore, the use of “push” messaging and social networks in a PSP may be confronted with “information overload” in which messages are not seen or not opened. The optimal frequency of messaging will depend on the disease, the treatment, the symptom burden and, of course, the patient’s personal preference. For example, adherence reminders should probably be issued on a daily basis for the at-home administration of SLIT but much less frequently for patients receiving SCIT. Another question is whether to introduce one technology-based intervention at a time or several simultaneously. A PSP must be able to anticipate and avoid “information fatigue” amongst its users. Lastly, messaging-based reminders may be unidirectional or bidirectional. In the latter situation, participants are encouraged to respond to reminders by giving information on adherence—even though this is usually impossible to verify. A smart, responsive system that takes account of the patient’s replies and redefines the messaging content accordingly may be preferable to “dumb”, alarm-clock-like reminders. Whereas poor adherence will generally trigger encouraging, advisory reminders, the opposite is also valid; congratulatory messages can be used to “reward” good compliance.
- *Custom platforms or open social media*? Mainstream social media platforms are easy to use and extremely wide-ranging but may not be sufficiently trusted and authenticated to convince and motivate patients. Validated, “official” sources of information should be developed in collaboration with patient associations and/or medical associations.
- *Age-specific content* Elderly adults, young adults, teenagers, young children and the latter’s parents have differing communication abilities, styles and habits. A PSP will have to be capable of using an appropriate language style when addressing a particular age group; communication will be totally different.
- *When in the patient’s journey can or should he/she be contacted by the PSP provider?* In AIT, it is probably best to initiate a PSP as soon as the patient has been diagnosed with an allergy because understanding the nature of allergic disease is essential for taking informed treatment decisions thereafter [48].
- *Interactivity and data validity* Should patients be able to request meetings or interactions with their physician or other health advisors? And if the PSP collects patient-reported data, will these data be reliable enough to be of use in setting or modifying the treatment strategy?
- *The involvement of “patient leaders”* It has been reported that patients with chronic conditions (heart disease, lung disease, stroke, or arthritis) benefit from short self-management courses in which they learn from other patients [49]. Furthermore, some countries have “train the trainers” courses for asthma, eczema or anaphylaxis; this could be extended to AIT.
- *Caregiver involvement* This is essential for pediatric PSPs and even for slightly older populations. For example, research in asthma has shown that caregiver support for adherence is still important in adolescence and young adulthood, even as these patients gain independence in dealing with their illness and treatment [50, 51].

## Conclusion

Multicomponent, multichannel, multistakeholder PSPs are needed to trigger patient engagement, increase knowledge about allergic diseases, overcome poor adherence to AIT and, ultimately, improve health outcomes through better patient self-management and stronger physician-patient partnerships which is of high importance especially in the field of AIT. By way of an analogy, the patient is no longer a mere “passenger”; the patient (and not the physician) is sitting in the driver’s seat, and the physician’s role is now to act as a guide and a coach. AIT providers have an important role to play (whether directly or indirectly) in PSPs, with a move towards this new paradigm.

The available evidence suggests that approaches with system-based reminders alone are not sufficiently effective on adherence. It would be interesting to design clinical trials in which adherence is the primary criterion, evaluating “hi-tech” interventions (based mainly on information technology) and “hi-touch” interventions (based mainly on interaction with humans, i.e. family members, patient mentors and healthcare professionals). However, the available evidence suggests that no single approach—whether tech- or human-based—has a significant, lasting impact on adherence; only “whole systems approaches” (combining patient-, provider and society-based actions) might do so [40].

## Abbreviations

AIT: allergy immunotherapy
PSP: patient support program
QoL: quality of life
SCIT: subcutaneous allergy immunotherapy
SLIT: sublingual allergy immunotherapy
